This article has been retracted.

# Encapsulation of Lactic Acid Bacteria by Lyophilisation with Its Effects on Viability and Adhesion Properties

**DOI:** 10.1155/2022/4651194

**Published:** 2022-05-27

**Authors:** Abhinandan Patil, Neha Munot, Mohsina Patwekar, Faheem Patwekar, Irfan Ahmad, Yasser Alraey, Saad Alghamdi, Ahmed Kabrah, Anas S. Dablool, Fahadul Islam

**Affiliations:** ^1^Sanjay Ghodawat University, Kolhapur, Maharastra, India; ^2^Vishwakarma University, Pune, Maharastra, India; ^3^Luqman College of Pharmacy, Gulbarga, Karnataka, India; ^4^Department of Clinical Laboratory Sciences, College of Applied Medical Sciences, King Khalid University, Abha, Saudi Arabia; ^5^Laboratory Medicine Department, Faculty of Applied Medical Sciences, Umm Al-Qura University, Makkah, Saudi Arabia; ^6^Department of Public Health, Health Sciences College, Al Leith, Umm Al-Qura University, Makkah, Saudi Arabia; ^7^Department of Pharmacy, Faculty of Allied Health Sciences, Daffodil International University, Dhaka 1207, Bangladesh

## Abstract

*Lactobacillus* (LAB) genera are considered important functional food but are found to have a short shelf life. In this study, two LAB, *Lactobacillus plantarum* (Lp) and *Lactobacillus rhamnosus* (Lr), were isolated from sheep's milk, and whole-genome sequencing was carried out by using 16s rRNA Illumina Nextseq, the Netherlands. The LAB were encapsulated by the lyophilisation technique using different lyoprotective pharmaceutical excipients. This process was carried out using a freeze dryer (U-TECH, Star Scientific Instruments, India). Shelf-life determination was carried out by a 12-month study using the viability survival factor (Vsf). The *in vitro* cell adhesion technique was carried out by using the red snapper fish along with autoaggregation and cell surface hydrophobicity as vital probiotic properties. It was observed that Lp has a significantly higher (*P* < 0.001) Vsf of 7.2, while Lr has a Vsf of 7 (*P* < 0.05) when both are encapsulated with 10% maltodextrin + 5% sucrose kept at 4°C for 12 months. The result demonstrated that Lp had significantly high (*P* < 0.05) cell adhesion, 96% ± 1.2 autoaggregation, and 6% cell surface hydrophobicity as compared to Lr. Moreover, this study demonstrated that lyophilised LAB with lyoprotective excipients enhances shelf life without any changes in probiotic properties when kept at 4°C exhibiting all its probiotic properties.

## 1. Introduction

Lactic acid bacteria are used for a long time as a functional food to treat many gastrointestinal-related disorders. *Lactobacillus* (LAB) genera are the most acceptable form of probiotics, obtained mostly from milk and milk products [1]. LAB are having a symbiotic association with the existing gastrointestinal microflora preventing dysbiosis and disease conditions. *Lactobacillus plantarum* (Lp) and *Lactobacillus rhamnosus* (Lr) are considered the most important lactic acid bacteria conferring health benefits [2]. Owing to their functional abilities, which means the desired pharmacological activities, nowadays, these probiotics are available in different formulation forms [3]. These formulation forms may be in tablets, capsules, and oral liquid monophasic single dosage forms. But the most concerning part is its short shelf life, as the formulation will prepare to deteriorate by a change in temperature and various storage conditions [4, 27–32]. Many studies revealed that the colony-forming unit (CFU) per gram value above 10^8^ counts is found to show the health benefits [5–10, 33]. But it is found that, during the storage condition, the CFU level falls below the threshold, resulting in zero pharmacological activities [11]. Thus, many drying techniques are employed to sustain the CFU g^−1^ value making it suitable for long-term storage [12].The spray drying method is found to be a most favourable technique to generate LAB granules. Spray drying yoghurt to preserve *Lactobacillus* and dairy starter cultures has been long investigated [13]. Lyophilised and spray-dried probiotic cultures are found to be stable with long-term storage life as compared to tray dry or other methods [14]. Yet, there are difficulties such as low survival rates of the probiotics during spray drying and poor rehydration properties of the resulting powders [15]. The final application of the food determines the type of microencapsulation and wall material to be used [16]. Freeze-dry or lyophilisation is another method to convert liquid LAB to dry powder form. Technological problems such as a sudden rise or fall in the temperature resulted in cell mortality or a decrease in the viability of LAB [17]. These problems are sorted by an introduction of many lyoprotective excipients [18]. Maltodextrin and lactose are the most preferred thermo-protective agents used in case of the spray dry method [19]. This excipient not only converts LAB into dry form but also maintains the viability for a long period.

Probiotic properties such as cell adhesion, autoaggregation, and hydrophobicity are found vital to fighting against pathogens. Cell adhesion of LAB was studied by many researchers using the fish intestine mucus model. Physiochemical abilities of the cell surface are hypothesized and are vital for cell adhesion in intestinal mucosa by means of hydrophobicity [20]. *In vitro* studies in LAB are investigated and proven to have preliminary potential to bind to the host cell [21]. Many investigators tried to find out the relationships between hydrophobicity and cell adhesion but failed to show the correlation between them [19, 25].

The present study deals with the encapsulation of the two different LAB isolated from sheep's milk. The aim is to evaluate the shelf life of LAB at two extremely different temperatures of 4°C and 37°C, to investigate the probiotic properties of LAB by hydrophobicity, cell adhesion, and autoaggregation methods, and furthermore, to determine if the encapsulation of LAB with different lyoprotective excipients affects the said probiotic properties and viability.

## 2. Materials and Methods

### 2.1. Isolation of Bacterial Strains and Its Cell Preparation

Two different probiotic nature lactic acid bacteria were isolated from sheep's milk samples using selective De Man, Rogosa, and Sharpe broth and agar media (MRS). This media was gifted as a free sample from Siffin Pharma, Germany [19, 22, 23]. These strains were identified as *Lactobacillus* by morphological and molecular identification using the 16s rRNA illumination Nextseq platform technique [24]. To generate the microbial load, these cells were grown in microaerophilic conditions using skim milk. All the cells were grown until the early stationary phase at 37°C for a period of 14 h until semisolid mass is formed. The semisolid mass generated was homogenised at 7500g for 10 min at 4°C using a REMI homogenizer. The liquid cell suspension was resuspended in different lyoprotective agents (w/v), i.e., 10% maltodextrin, 10% lactose, 10% sucrose, 10% maltodextrin + 5% sucrose, and 10% lactose + 5% sucrose prior to lyophilisation, where skim milk was kept as the control.

### 2.2. Lyophilisation and Storage

The cell suspension prepared was added into sterile vials. The vials were frozen at −20°C overnight in a freeze dryer (U-TECH, Star Scientific Instruments, India). Furthermore, the vials were incubated at −70°C for 1 h and late freeze-dried at −50°C at 110 millitorr chamber pressure of a condenser for 48 h [24].

The cells obtained were dried and packed in a plastic container at 4°C, i.e., refrigeration at 37°C (room temperature) under Indian climatic conditions for a period of 12 months.

### 2.3. Cell Viability Determination

The cell viability was determined by the serial dilution technique on the MRS media. The cell count of the prepared sample before lyophilisation and after encapsulation was determined by the CFU count [25]. Both types of the sample, i.e., before and after lyophilization, were rehydrated in a 1 ml solution of 5% dextrose aliquot for 20 min at 37°C with gentle shaking. The above-said samples were plated on the MRS media at 37°C for a period of 24 h in microaerophilic conditions [20]. The cell viability during the long-term storage for 12 months was expressed as the viability storage factor (Vsf). This calculation of Vsf was performed as Vsf = 1 (log CFU0 – log CFUX)/log CFUX *X* 10, where CFU0 = initial CFU g-1 X total weight of the dry sample (g), while CFUX = *X* (0, 1, 2,… N value in hours) time CFU g-1 X weight of the dry sample (*g*). The calculation was multiplied by 10 to get the value of Vsf in integrals and to avoid the values in decimals.

### 2.4. Probiotic Properties of *Lactobacillus*

Various probiotic properties such as the degree of surface hydrophobicity and the cell autoaggregation nature were investigated. This includes the results after the lyophilisation process and during the storage condition.

### 2.5. *In Vitro* Cell Adhesion Techniques Using Red Snapper

Red snapper fish were purchased from a local market near sea coastal areas of Ratnagiri, India. These fishes were strived for 24 h and were sacrificed. The intestine of the fish was transferred to the Petri dish, and mucus was removed by scrapping the mucosal surface [20]. The mucus was then homogenised and centrifuged at 8000g for 15 min at 4°C to remove other cellular debris. Finally, the mucus suspension was sterilised in UV light and stored in an aseptic container at −20°C. Later, 100 *µ*l of the LAB was added into the 200 *µ*l solution of freshly prepared mucus suspension previously coated on the microtiter plate wells. Furthermore, the LAB cells were incubated for 1 h at 37°C with the mucus suspension. The incubated suspension was washed thrice with saline solution to remove the nonadherent cells. The suspension was kept at 60 ^0^C for 15 min and was stained with 0.5% crystal violet for 45 min [22]. The excess stain was removed by saline solution wash, and absorbance was taken at 640 nm using a microtiter plate reader. Mucus stained without LAB was considered as the control and by subtracting these values of the control, the final absorbance values were recorded.

### 2.6. Autoaggregation Assay

This assay was performed by incubating the two different LAB strains in MRS broth at 37°C for 24 h. The cells were centrifuged at 4000 g for 20 min initially by maintaining the cell count at 10^8^ CFU/mL [20]. The cell suspension of 4 mL, after vortexing for 20 sec, helped to determine the autoaggregation activity every hour for a period of 5 h incubated at 25°C. Generally, at the period of 1 h, 0.1 mL of the superficial suspension was transferred to 3.9 mL of phosphate buffer solution (PBS) of pH 7.4 measured at 620 nm absorbance.

The autoaggregation (Aa) was determined and calculated as Aa= (1-Ax/A0) *X* 100, where *x* denotes time interval in hours and A0 denotes absorbance at time *t* = 0.

### 2.7. Determination of Cell Surface Hydrophobicity

The cells were incubated in MRS broth at 37°C for a period of 24 h. Later, the cells were washed with PBS, and the optical density was adjusted at 0.5 ± 0.01 at 450 nm [26]. 60 *µ*l of xylene was added to 1 mL of cell suspension after vortexing for 1 min. The optical density of the water from biphase is determined as percentage (%) hydrophobicity = (1−AA/AB) *×* 100, where the optical density values are calculated as AA (after) and AB (before).

### 2.8. Scanning Electron Microscopy Study of Encapsulated Lactic Acid Bacteria

Both the encapsulated LAB were observed by scanning electron microscopy, in which the size of the particles was evaluated.

### 2.9. Statistical Analysis

Dunnett's multiple comparison tests of ANOVA were used to compare the values of each parameter of the LAB. GraphPad Prism 5.01 (GraphPad Software, Inc., USA) software was used for basic analysis and graphical data interpretation. Experiments were carried out in triplicate with a level of significance for all analyses determined at *P* < 0.05, 0.01, 0.001.

## 3. Results and Discussion

### 3.1. Viability Study of *Lactobacillus* during Lyophilisation

Two different strains of bacteria, isolated from sheep's milk were identified as LAB, i.e*., Lactobacillus rhamnosus* (Lr) and *Lactobacillus plantarum* (Lp) by morphological and molecular analysis by 16s rRNA identification. The LAB which grew on MRS media was with small, circular, white-creamy color, and nontransparent colonies proved by morphological characters as shown in Figure 1. Microscopically both the isolates were Gram-positive, rod-shaped, nonmotile, catalase-negative, and lacked endospores. Patil et al. observed the same morphological characteristics such as the Gram staining and plating methodology along with the serial dilution method [19]. Both the LAB strains were analysed for resistance during lyophilisation using different lyoprotective excipients. The LAB strain Lr showed CFU mL^−1^ values higher in 10% maltodextrin + 5% sucrose and 10% lactose + 5% sucrose, i.e., 9.4 ± 0.22, 8.9 ± 0.15 before and 9.1 ± 0.18, and 8.6 ± 0.14 after encapsulation. However, in the case of Lp, the CFU mL^−1^ values found were 9.5 ± 0.05, 9.1 ± 0.21 before, and 9.1 ± 0.16, 8.4 ± 0.21 after lyophilisation (Table 1). During encapsulation, very negligible changes in the CFU g^−1^ count were observed in the case of both the LAB samples. Thus, for ease in understanding the role of lyoprotective excipients, the CFU g^−1^ values found in the case of skim milk were kept as the control with values 7.2 ± 0.14, 7.2 ± 0.14 before, and 6.0 ± 21, 6.2 ± 0.16 after lyophilisation in the case of Lr and Lp, respectively. The values noted for 10% sucrose as an excipient were found with the least CFU g^−1^ count with 8.2 ± 0.24, 8.1 ± 0.14 before and 7.4 ± 0.22, 6.5 ± 0.17 values after lyophilisation for Lr and Lp, respectively (Table 1). According to Abd-Talib et al., different excipients such as gelatin and maltodextrin play an important role in the cell survival rate. In this study, he has shown the reduced cell viability from 3.25 × 10^7^ CFU mL^−1^ to 2.15 × 10^7^ CFU mL^−1^ during a two-week study [15]. He also described that the viability of the LAB depends on the excipients used for the drying technique. Thus, the same kind of results were observed in the LAB lyophilisation process showing the importance of different lyoprotective excipients and their effects on the viability count.

### 3.2. Viability Studies of *Lactobacillus* during Storage

Comparative studies were carried out in the case of two LAB strains for long-term stability testing. The lyophilised products were screened for a period of 12 months under two different extreme conditions, i.e., at 4°C and at 37°C. In the case of all strains, a significantly higher survival (*P* < 0.05) rate was found at 4°C as compared to 37°C. During the study, a skim milk lyophilised product was considered as the control. This control group was compared with the rest of the other lyoprotective excipient combination groups. In the case of the Lr group at 4°C, the 10% maltodextrin +5% sucrose group shows a significantly higher survival rate, i.e., a Vsf value of 7.8 (*P* < 0.05) as compared to the control group after 12 months of studies, as shown in Figure 2(a). While in the case of the Lp group at 4°C, the 10% maltodextrin°+°5% sucrose group shows highly significant survival (*P* < 0.001) as compared to the control group with the Vsf value around 7.2. Similarly, the 10% maltodextrin group shows a significantly high survival count (*P* < 0.01) as compared to the control group with a Vsf value of 6.2 after a 12-month study. The 10% sucrose group shows a significantly high survival rate (*P* < 0.05) with a Vsf value of 5.1 when the study was conducted for the period of 12 months as seen in Figure 2(b). On the contrary, the 10% lactose group and 10% lactose + 5% sucrose group did not show any significant (*P* < 0.05) survival range as compared to the control group.

When the same Vsf study was determined at 37°C temperature, it was found that no survival count found after 6 months of tenure was analysed by the serial dilution technique. In the case of the Lr group at 37°C temperature shelf-life study, the 10% maltodextrin + 5% sucrose group showed the highest significant survival (*P* < 0.001) count as compared to the control group with a Vsf value of 3.1 after 6 months of study as seen in Figure 3(a). However, the 10% lactose + 5% sucrose group shows a significantly higher survival rate (*P* < 0.01) with a Vsf value of 2.9 after a 6-month study. Similarly, the 10% maltodextrin group shows a significantly high Vsf value, i.e., 2.5 after 6 months of study as compared to the control group.

In a similar type of study, when carried out in the case of Lp at 37°C, significantly variable results were obtained (*P* < 0.05) for 6 months of study. In the case of Lp at 37°C, the 10% maltodextrin + 5% sucrose group shows a significantly higher (*P* < 0.01) Vsf value, i.e., 3.0, after a 6-month long-term study as compared to the control group as shown in Figure 3(b). Similarly, the 10% lactose + 5% sucrose group shows a significantly high (*P* < 0.05) Vsf value, i.e., 2.2 as compared to the control. T. Ozcan et al. described that, in fermented beverages of *L. rhamnosus* in apples and blueberries, the growth of probiotic bacteria is influenced by the physicochemical properties of the media along and storage conditions at refrigeration [3]. They showed the same results by short-term refrigeration based on the Viability and Growth Proportion Index (GPI) of the LAB. According to their study, *L. rhamnosus* showed significantly higher viability and GPI than *L. acidophilus* in all conditioned natural media they generated.

### 3.3. *In Vitro* Red Snapper Fish Assay

In case of adherence abilities of LAB isolates, Lp and Lr were tested in the red snapper fish's intestinal mucus. The result showed that Lp adhered (*P* < 0.05) significantly higher (OD_640_ = 0.60 ± 0.83) than Lr (OD_640_ = 0.31 ± 0.93). No significant difference was observed in the case of adherence properties of Lp and Lr after lyophilisation by using the different lyoprotective excipients as shown in Figure 4. It was found that lipoteichoic acids were the responsible factor for adhesion in the LAB [21]. Similarly, various adhesion proteins responsible for cell autoaggregation and adhesion were previously studied in the LAB [22]. Thus, a similar kind of adhesion process is demonstrated in Lp and Lr. Georgia Saxami et al. studied the adhesion properties of *L. pentosus* and *L. plantarum*, isolated from table olives. They demonstrated that both strains exhibited higher adhesion rates to CaCO_2_ colon cancer cells and compared that with the control group of *L. casei.*

### 3.4. Autoaggregation

The autoaggregation phenomenon was observed by the phenotypic technique. Lp in all forms after lyophilisation showed 96 ± 1.4% of autoaggregation. Similarly, Lr in all forms showed 91% ± 2.1 autoaggregation analysed by the formation of the precipitate and turbid solution formation (Table 2). This similar type of work was observed in the case of *Clostridium butyrium* broth showing precipitate even after a wash with PBS solution [23]. The autoaggregation helps the LAB to prevent the adhesion of pathogenic microbes to gastrointestinal mucus.

### 3.5. Hydrophobicity Analysis of Cell Surface

A hydrophobicity study was conducted to determine the relationship between mucosal adhesion by the LAB and its physiochemical properties. Lp showed 6.2 ± 1.51% cell surface hydrophobicity; similar results were observed in the case of Lp with its different lyoprotective excipient combinations. Significantly, no difference in hydrophobicity was observed in the case of Lr as it showed 7.2 ± 0.51% along with its other excipient combinations (Table 2). Vinderola et al. tried to find such a relationship between adhesion and hydrophobicity, but none of them were successful [23]. The same results were observed in the case of both LAB, thus not showing any relationship between hydrophobicity and adhesion abilities.

### 3.6. Particle Size Determination

The SEM method proved that the granule obtained is in a spherical form with a dimension of 4.8 to 5.42 *µ*m in the case of *Lactobacillus plantarum* as shown in Figure 5(a) and *Lactobacillus rhamnosus* as shown in Figure 5(b).

## 4. Conclusion

The current study demonstrated lyophilisation of LAB isolated from sheep's milk. The study conducted proves that the highest resistance was observed during the drying process by using 10% maltodextrin + 5% sucrose as compared to other lyoprotective excipients which were used for the excipient during all processes. The selected excipient (10% maltodextrin + 5% sucrose) ratio shows a significantly high survival rate in the case of both LAB kept at 4°C condition for a 12-month study. *Lactobacillus plantarum* showed significantly higher probiotic properties such as *in vitro* adhesion, autoaggregation, and hydrophobicity as compared to *Lactobacillus rhamnosus* which was conducted by the red snapper fish assay. Both the lyophilised LAB by different lyoprotective excipients did not show any change in probiotic properties after encapsulation.

Finally, it is proved that lyophilised *Lactobacillus plantarum* and *Lactobacillus rhamnosus* show good viability and survival nature when stored at 4°C for 12 months as compared to a room temperature of 37°C.

## Figures and Tables

**Figure 1:** The lactic acid bacteria on MRS media with serial dilution and morphological characteristics. (a) Colonies of *Lactobacillus rhamnosus* were circular pinpoint and white uniform-sized. (b) Colonies of *Lactobacillus plantarum* were circular blunt, with entire elevated margin.

**Figure 2:** Shelf life of lyophilised LAB strain. (a) *Lactobacillus rhamnosus* at 4°C and (b) *Lactobacillus plantarum* at 4°C with different lyoprotective agents (w/v), i.e., 10% maltodextrin, 10% lactose, 10% sucrose, 10% maltodextrin + 5% sucrose, and 10% lactose + 5% sucrose, where skim milk was kept as control. Values presented are the means and standard deviations from three replicates. ^*∗∗∗*^(*P* < 0.001), ^*∗∗*^(*P* < 0.01), ^*∗*^(*P* < 0.05).

**Figure 3:** Shelf life of lyophilised LAB strain. (a) *Lactobacillus rhamnosus* at 37°C and (b) *Lactobacillus plantarum* at 37°C, with different lyoprotective agents (w/v), i.e., 10% maltodextrin, 10% lactose, 10% sucrose, 10% maltodextrin + 5% sucrose, and 10% lactose + 5% sucrose, where skim milk was kept as control. Values presented are the means and standard deviations from three replicates. ^*∗∗∗*^(*P* < 0.001), ^*∗∗*^(*P* < 0.01), ^*∗*^(*P* < 0.05).

**Figure 4:** Adhesion assay of LAB strain including both *Lactobacillus rhamnosus* and *Lactobacillus plantarum* with different lyoprotective agents (w/v), i.e., skim milk, 10% maltodextrin, 10% lactose, 10% sucrose, 10% maltodextrin + 5% sucrose, and 10% lactose + 5% sucrose. Values presented are the means and standard deviations from three replicates.

**Figure 5:** Scanning electron microscopic images of (a) *Lactobacillus plantarum* and (b) *Lactobacillus rhamnosus* with its dimensions.

**Table 1:** Lyophilisation of LAB with the excipients and its CFU mL^−1^ count.

LAB	Excipient ratio	Log CFU mL^−1^ (^*∗*^×10^9^)^a^	
		Before L	After L
*Lactobacillus rhamnosus*	Skim milk	7.2 ± 0.14	6.0 ± 0.21
	10% sucrose	8.2 ± 0.24	7.4 ± 0.22
	10% maltodextrin	9.1 ± 0.36	8.9 ± 0.27
	10% lactose	8.8 ± 0.17	8.2 ± 0.13
	10% maltodextrin and 5% sucrose	9.4 ± 0.22	9.1 ± 0.18
	10% lactose and 5% sucrose	8.9 ± 0.15	8.6 ± 0.14

*Lactobacillus plantarum*	Skim milk	7.2 ± 0.24	6.2 ± 0.16
	10% sucrose	8.1 ± 0.22	6.5 ± 0.17
	10% maltodextrin	9.2 ± 0.27	8.4 ± 0.12
	10% lactose	8.6 ± 0.34	8.1 ± 0.18
	10% maltodextrin and 5% sucrose	9.5 ± 0.05	9.1 ± 0.16
	10% lactose and 5% sucrose	9.1 ± 0.21	8.4 ± 0.21

a: survival is described as the mean of the log CFU mL^−1^, *n* = 3; b: yield represented the mean of percentages of product obtained; ±: the standard error of the mean; L^*∗*^: lyophilisation method (*p* < 0.05).

**Table 2:** Percentage of hydrophobicity and autoaggregation of LAB.

Bacterial isolates	Excipient combination	% autoaggregation	% cell-surface hydrophobicity
*Lactobacillus rhamnosus*	Skim milk	91 ± 1.5	7.2 ± 1.51
	10% sucrose	90 ± 1.7	7.0 ± 0.56
	10% maltodextrin	91 ± 2.4	6.9 ± 1.21
	10% lactose	90 ± 1.4	7.1 ± 1.54
	10% maltodextrin and 5% sucrose	91 ± 2.1	7.2 ± 1.15

*Lactobacillus plantarum*	10% lactose and 5% sucrose	90 ± 1.1	6.9 ± 1.42
	Skim milk	96 ± 1.4	5.9 ± 1.42
	10% sucrose	96 ± 2.4	6.1 ± 1.12
	10% maltodextrin	96 ± 1.8	6.0 ± 1.42
	10% lactose	96 ± 2.2	6.0 ± 1.52
	10% maltodextrin and 5% sucrose	96 ± 1.7	6.0 ± 1.16
	10% lactose and 5% sucrose	96 ± 0.8	6.0 ± 1.05

a: Survival is described as the mean of the log cfu mL^−1^, n = 3; b: Yield represented as the mean of percentages of product obtained, ± the standard error of the mean.; L^∗^- Lyophilisation method (*p* < 0.05).

## Data Availability

All data used to support the findings of this study are included within the article.
